The article "Gaucher’s Disease in an Adult Male: A Case Report of a Rare Mutation" was published in 2024. Journal: Cureus.

# Gaucher’s Disease in an Adult Male: A Case Report of a Rare Mutation

**DOI:** 10.7759/cureus.58706

**Published:** 2024-04-22

**Authors:** Adityasinh A Bhati, Smit R Shah, Yagnya D Dalal, Nehal M Shah, Monila N Patel

**Affiliations:** 1 Internal Medicine, Smt. Nathiba Hargovandas Lakhmichand (NHL) Municipal Medical College, Ahmedabad, IND; 2 Medicine, GCS Medical College, Ahmedabad, IND

**Keywords:** pancytopenia, bone marrow biopsy, gene mutation, hepatosplenomegaly, gaucher's disease

## Abstract

Gaucher’s disease is a rare autosomal recessive inborn error of metabolism. As the presentation of this disease is similar to more common diseases like malaria, portal hypertension, hematological disorders, and kala-azar, this rare disease may not be thought of as a differential diagnosis, and a high index of suspicion is required to avoid diagnostic delay. We report a case of type 1 Gaucher’s disease in an adult male born out of a consanguineous marriage. He was from a region where the prevalence of infectious diseases and sickle cell anemia is high. He presented with abdominal distension, hepatosplenomegaly, and pancytopenia. Bone marrow biopsy showed the presence of Gaucher cells. Glucocerebrosidase levels showed decreased enzyme activity. The genetic study revealed a very rare mutation that has not been reported in the 1000 Genomes database till now. Retrospectively, the most important clue was his birth out of a consanguineous marriage of his parents.

## Introduction

Gaucher’s disease is a rare, autosomal recessive, metabolic disorder caused by mutations in the glucocerebrosidase (GBA1) gene [1]. This causes beta-glucocerebrosidase enzyme deficiency, leading to the toxic accumulation of glucocerebroside lipids in various tissues in the body [1,2]. Most commonly, they are accumulated in the spleen, liver, and bone marrow. Gaucher’s disease mainly presents in childhood, and half of the patients are diagnosed before the age of 10 years [3]. As Gaucher's disease is an autosomal recessive disorder, it affects males and females both. The male:female ratio is 0.85:1 [3]. This case highlights the challenges of diagnosing Gaucher’s disease in adults, particularly in regions with a high prevalence of infectious diseases with similar symptoms. This case also emphasizes the importance of accessible screening for Gaucher’s disease, especially in populations with high rates of consanguineous marriages.

## Case presentation

A 39-year-old Indian Muslim male patient born out of a consanguineous marriage presented with complaints of abdominal distension for 10 months, low-grade intermittent fever, anorexia, and weight loss. The fever was relieved by non-steroidal anti-inflammatory drugs (NSAIDs) and was not associated with chills or rigors. There were no associated complaints of abdominal pain, nausea, vomiting, diarrhea, constipation, or bone pain. He had a history of jaundice at the age of 18 years, which had relieved on its own, and no documents were available for that episode. He had a normal birth and developmental history. His parents did not have similar health problems. He had one sister and four brothers. None of them ever had any significant health problems. He had no history of addiction or substance abuse.

The article "Gaucher’s Disease in an Adult Male: A Case Report of a Rare Mutation" was published in 2024. Journal: Cureus.

On examination, the patient had pallor and icterus. The abdomen was distended and globular in shape with an everted umbilicus (Figure 1). The liver was enlarged up to 10 cm below the right costal margin. The spleen was enlarged crossing the midline and reaching up to the right iliac fossa. There were no signs of free fluid in the abdomen. Neurological and skeletal system examination was normal.

**Figure 1:** Abdominal distension with everted umbilicus

Lab investigations are presented in Table 1. The patient had pancytopenia. Sputum, urine, and blood cultures were negative.

**Table 1:** Relevant laboratory investigations WBC: white blood cell, SGPT: serum glutamic-pyruvic transaminase, SGOT: serum glutamic-oxaloacetic transaminase, TIBC: total iron binding capacity, PT: prothrombin time, INR: international normalized ratio, aPTT: activated partial thromboplastin time, LDH: lactate dehydrogenase

Test	Patient value	Reference value
Hemoglobin (g/dL)	6.1	14-18
WBC (/mm^3^)	1300	4000-11,000
Platelets (/mm^3^)	25000	1,50,000-4,00,000
SGPT (U/L)	30	7-56
SGOT (U/L)	112	8-45
Bilirubin total (mg/dL)	6.68	0.1-1.2
Bilirubin direct (mg/dL)	2.97	<0.3
Bilirubin indirect (mg/dL)	3.71	0.2-0.8
PT (seconds)	52	11-13.5
INR	2.5	0.8-1.1
aPTT (seconds)	48.4	21-35
Total S. protein (g/dL)	6.68	6-8.3
S. albumin (g/dL)	2.97	3.4-5.4
S. calcium (mg/dL)	8.1	8.5-10.2
Iron (mcg/dL)	14	70-175
Ferritin (ng/mL)	>1650	12-300
TIBC (mcg/dL)	270	240-450
Reticulocyte count	0.8%	0.5-2.5%
LDH (U/L)	275	140-280
Lipid profile, renal function test, urine examination	Normal	
Anti-nuclear antibodies (ANA), HIV (rapid test), HB_s_Ag, anti-HCV antibodies, malarial parasites	Negative	

The fundoscopic examination was normal. Abdominal ultrasonography showed hepatomegaly measuring 20 cm in its long axis with altered echotexture and irregular margin, suggestive of liver parenchymal disease. It showed splenomegaly measuring 24 cm in its long axis and showed multiple mixed echogenic lesions with hypoechoic perilesional rim without internal vascularity. Splenic lesions were suggestive of developing abscesses. Liver FibroScan was suggestive of mild fibrosis. His ECG and echocardiogram were normal.

The article "Gaucher’s Disease in an Adult Male: A Case Report of a Rare Mutation" was published in 2024. Journal: Cureus.

To investigate the cause of massive hepatosplenomegaly in a background of pancytopenia, a bone marrow biopsy was done (Figure 2). It showed the presence of clusters and sheets of large macrophages containing a small nucleus and abundant pale, fibrillary cytoplasm resembling wrinkled tissue paper appearance, which is replacing hematopoietic tissues. Reserved hematopoietic tissues showed mild hyperplasia of erythroid precursors and megakaryocytic cells. The findings were suggestive of Gaucher’s disease.

**Figure 2:** Histopathology of bone marrow biopsy Arrow showing large macrophage containing a small nucleus and abundant pale, fibrillary cytoplasm resembling wrinkled tissue paper appearance suggestive of a Gaucher cell.

Beta-glucosidase levels were tested, which was suggestive of a deficient state: 2.4 nmol/hr/mg protein (normal range: 4.0-32.0 nmol/hr/mg protein). Plasma chitotriosidase levels were elevated: 16052.3 nmol/hr/mg protein (normal range: 28.66-62.94 nmol/hr/mg protein). A genetic study done by sm-MIP (molecular inversion probe) and NGS detected the presence of a homozygous variant for c.1184C>T (p.Ser395Phe) in exon-8 of the GBA gene, confirming the diagnosis of Gaucher’s disease. This variant has not been reported in the 1000 Genomes database and has a minor allele frequency (MAF) of 0.0008% in the gnomAD database.

The patient was advised on enzyme replacement therapy. However, he could not afford the cost of the treatment. Some nongovernmental organizations (NGOs) were requested to provide financial aid to the patient.

## Discussion

Among the lysosomal storage disorders, Gaucher’s disease is the most common disorder with 1/40,000 prevalence [4]. The relatively higher prevalence is seen in the Ashkenazi Jewish population, which is roughly around 1/1000, with one in 10 carriers [5]. As Gaucher’s disease is rare, the actual prevalence of the disease is understated. A low level of clinical suspicion on the physician’s part leads to the underdiagnosis of the disease. Among Indians, Gaucher’s disease is more prevalent in the Parsi community with its prevalence being as high as 1/2500 to 1/5000. The GBA gene is located on chromosome 1q21, and its mutation leads to the deficiency of the glucocerebrosidase enzyme. Among more than 300 mutations documented in Gaucher’s disease, L444p is most common in India [6]. Our patient has the presence of a very rare homozygous variant, which has not been reported in the 1000 Genomes database and has an MAF of 0.0008% in the gnomAD database.

Gaucher’s disease is mainly classified into three types based on the age of onset, neurological involvement, and severity. These types are type 1 (non-neuronopathic, chronic/adult form), type 2 (acute neuropathic, acute/infantile form), and type 3 (subacute neuropathic, subacute/juvenile form). Type 1 is the most common and milder form of Gaucher’s disease. It is characterized by a lack of neurological symptoms. More than half of the patients are diagnosed before the age of 20 years. Patients usually have hepatomegaly, massive splenomegaly, pancytopenia, bone involvement, and failure to thrive. Lung involvement in the form of diffuse infiltration may occur. In adults, pulmonary hypertension has been documented in splenectomised patients rarely [7]. Patients usually have normal life expectancy, but conditions like non-Hodgkin's lymphoma, multiple myeloma, Parkinsonism, and peripheral neuropathy are associated with it [7]. Our patient belonged to this category. Type 2 is the most severe form of the disease, characterized by severe neurological symptoms and a rapid decline in neurological function. The age of onset is before two years. It has a rapidly progressive course and patients usually die by two to four years of age. Patients have neurological manifestations in the form of pyramidal signs (retroflection of the head, opisthotonus, spasticity, and trismus) and bulbar signs (squint, stridor, and feeding difficulty) in addition to classic multi-system involvement [8]. Type 3 is relatively more common in India compared to the Western countries. The mean age of onset is five years, and the mean age of neurological involvement is eight years. This form is intermediate in severity between type 1 and type 2 of Gaucher’s disease. Patients with type 3 disease have a slowly progressive course as compared to type 2 disease with a life span extending up to the fourth decade of life. Patients have varied presentations with supranuclear saccadic horizontal gaze palsy, nystagmus, developmental delay, hearing impairment, generalized tonic-clonic seizures, progressive myoclonic seizures, dementia, and ataxia [9].

The article "Gaucher’s Disease in an Adult Male: A Case Report of a Rare Mutation" was published in 2024. Journal: Cureus.

Other rare variants of Gaucher’s disease are the perinatal lethal form and the cardiovascular form. The perinatal lethal form is a rare variant having severe manifestations in uteri or at birth presenting as collodion baby, hydrops fetalis, hepatosplenomegaly, and ascites. Arthrogryposis and dysmorphic facial features can be noted in up to 40% of cases [10]. The cardiovascular form is a rare variant that has predominant cardiac involvement in the form of aortic and mitral valve calcification [11]. Additional findings include corneal opacities, splenomegaly, and ophthalmoplegia.

Management of Gaucher’s disease includes a multidisciplinary approach. Specific modalities include enzyme replacement therapy (ERT), substrate reduction therapy (SRT), and bone marrow transplant. Supportive management options include correction of anemia, vitamin D supplements, bisphosphonates, and splenectomy [12]. ERT has been effective in reducing organomegaly. It also helps reduce the problems caused by bone involvement. However, the ERT is not effective in reducing neurological symptoms because the enzyme does not cross the blood-brain barrier. SRT acts by reducing the formation of substrate precursor to a level so that it can be handled by low levels of the enzyme.

## Conclusions

This case report highlights the challenges of diagnosing Gaucher’s disease in adults presenting with similar symptoms like infectious diseases, hemoglobinopathies, leukemia/lymphoma, and portal hypertension particularly in developing countries like India. This case emphasizes the importance of clinical suspicion on the part of clinicians and the requirement of accessible screening for Gaucher’s disease, especially in populations with high rates of consanguineous marriages. Furthermore, the identification of a rare homozygous variant in this patient underscores the need for more data and research on Gaucher’s disease in developing countries. The genetic makeup of Gaucher’s disease patients in India might be significantly different from the Western population. Further research is crucial to understand the specific spectrum of Gaucher’s disease mutations and their clinical manifestations in developing countries.
